# Production Optimization and Biochemical Characterization of Cellulase from *Geobacillus* sp. KP43 Isolated from Hot Spring Water of Nepal

**DOI:** 10.1155/2022/6840409

**Published:** 2022-05-12

**Authors:** Subash Khadka, Deegendra Khadka, Ram Chandra Poudel, Mukund Bhandari, Purnima Baidya, Jaishree Sijapati, Jyoti Maharjan

**Affiliations:** ^1^Molecular Biotechnology Unit, Nepal Academy of Science and Technology, Lalitpur, Nepal; ^2^Central Department of Microbiology, Tribhuvan University, Kathmandu, Nepal; ^3^Department of Molecular Medicine, University of Texas Health Science Center at San Antonio, Texas, USA; ^4^Department of Population Health Sciences, University of Texas Health Science Center at San Antonio, Texas, USA

## Abstract

This study is aimed at isolating and identifying a thermophilic cellulolytic bacterium from hot spring water and characterizing thermostable cellulase produced by the isolate. Enrichment and culture of water sample was used for isolation of bacterial strains and an isolate with highest cellulase activity was chosen for the production, partial purification, and biochemical characterization of the enzyme. Different staining techniques, enzymatic tests, and 16s ribosomal DNA (16s rDNA) gene sequencing were used for the identification of the isolate. The cellulase producing isolate was Gram positive, motile, and sporulated rod-shaped bacterium growing optimally between 55°C and 65°C. Based on partial 16s rDNA sequence analysis, the isolate was identified as *Geobacillus* sp. and was designated as *Geobacillus* sp. KP43. The cellulase enzyme production condition was optimized, and the product was partially purified and biochemically characterized. Optimum cellulase production was observed in 1% carboxymethyl cellulose (CMC) at 55°C. The molecular weight of the enzyme was found to be approximately 66 kDa on 12% SDS-PAGE analysis. Biochemical characterization of partially purified enzyme revealed the temperature optimum of 70°C and activity over a wide pH range. Further, cellulase activity was markedly stimulated by metal ion Fe^2+.^ Apart from cellulases, the isolate also depicted good xylanase, cellobiase, and amylase activities. Thermophilic growth with a variety of extracellular enzyme activities at elevated temperature as well as in a wide pH range showed that the isolated bacteria, *Geobacillus* sp. KP43, can withstand the harsh environmental condition, which makes this organism suitable for enzyme production for various biotechnological and industrial applications.

## 1. Introduction

Microbial life does not seem to be limited to specific environments as microbial communities can be found in most diverse conditions including extreme temperature, pressure, pH, and salinity, which are referred as extremophiles [1, 2]. Survival of microorganisms in extreme environments requires the production of enzymes that function under those conditions. Realizing this fact, industries have been fueling research on novel enzymes from extremophiles including thermophiles to use them as catalysts [3]. Thermophiles are group of microorganisms that grow at a temperature between 55°C and 85°C [4]. Thermostable enzymes, such as *α*-amylase, cellulase, *α*-glucosidase, *α*-galactosidase, *β*-glucosidase, *β*-galactosidase, protease, pullulanase, and xylanase, can be obtained from thermophilic organisms [5]. Thermostable enzymes are much advantageous to industrial processes because of accelerating reaction rate, improving substrate solubility, ameliorating solvent miscibility, and lessening the risk of contamination of a system at a high temperature [6]. So, thermophilic organisms have received the attention mostly due to the stability of their enzymes at elevated temperatures, which is often required in biotechnological processes.

With increased industrialization combined with the fact that cellulose is the most abundant renewable raw material and energy source, cellulases have found a wide range of application in numerous industries such as agriculture, pulp and paper, textile, food and beverage, animal feed, and detergent and also in bioconversion of cellulosic material into solvents such as ethanol [7]. Extensive use of fossil fuels and resulting CO_2_ accumulation is a major cause of global warming [8]. This situation forced many countries in the world to explore new possibilities for biogas, bioethanol, biodiesel, and fuel cell production from renewable resources [9]. Ethanol blended fuel in automobiles significantly reduces petroleum use and greenhouse gas emission [10].

Hydrolysis of cellulose present in lignocellulosic biomass to produce reducing sugars and their subsequent fermentation are essential steps for production of ethanol. This conversion of cellulose to sugars occurs more rapidly at elevated temperatures as cellulose swells at these temperatures facilitating rapid degradation [11]. This highlights that thermostability is a major requirement for efficient hydrolysis of cellulose by cellulases. Known cellulases from nature cannot function at temperatures higher than about 50°C [11] at which bioconversion is slow with higher risk of contamination. Since thermostable enzymes last longer at higher temperatures, this translates to more cellulose being broken down thereby reducing the cost of production. Consequently, there is an increasing demand for stable, highly active, and specific cellulases at a minimal cost [12].

This study targets hot springs for bioprospecting thermophilic bacteria as they make a potential source of extremophiles [13]. Although more than 28 hot springs are reported in Nepal [14], their microbial diversity and hence the biotechnological potential of those microbes await exploration in detail [15]. Research on microbes with bioconversion potential is of more importance in countries like Nepal, where agriculture-based industries generate tons of lignocellulosic waste, but these resources are not being utilized efficiently. Utilization of such resources for production of renewable energy (bioethanol) has dual advantages for Nepal: (i) reduced import of fossil fuels and (ii) economical management of agricultural wastes. Moreover, every little step taken to produce bioethanol economically might slowly discourage the massive dependence on fossil fuels making the world healthier place for living by stepping toward renewable energy production era. Realizing this fact, the present study is aimed at characterizing extracellular thermophilic cellulase produced by *Geobacillus* sp. KP43. To our knowledge, this is the first report describing the production of thermoalkalophilic cellulase by *Geobacillus* sp. KP43 isolated from Kharpani hot spring.

## 2. Materials and Methods

### 2.1. Sample Collection

Water sample was collected in a sterile plastic bottle from “Kharpani hot spring” (altitude 1238 m, latitude 28°21′39.9^″^ N and longitude 83°57′37.5^″^ E) located on the bank of the Seti river, 21 km north from Pokhara, Nepal. The temperature and pH of the spring were noted to be 69.5°C and 6.19, respectively. The sterile collection bottle was filled with pooled water sample from three different locations of the spring close to the center, capped tightly, and transported to the laboratory of Nepal Academy of Science and Technology (NAST), Kathmandu, Nepal.

### 2.2. Isolation of Bacterial Strains

A total of 44 bacterial strains were isolated by enrichment of the water sample on Nutrient Broth (NB) at 60°C followed by subculture to Nutrient Agar (NA) plates. Each distinct and isolated colony was transferred to fresh agar plates repeatedly to ensure purity of the isolate. Each isolate was preserved as a glycerol stock at -80°C for future use.

### 2.3. Screening of Isolates for Extracellular Enzyme Production

Cellulase enzyme was screened by growing the isolates for 24 hours at 60°C in a basal cellulose agar medium containing 2% agar, different salts, and 0.5% carboxymethyl cellulose (CMC) as only carbon source [16]. The cellulolytic ability of each isolate was screened by flooding the plates with Lugol's iodine [17] and also by sequential flooding of 1% Congo red and 1 M NaCl [18]. The ability of the isolate to hydrolyze substrates other than cellulose (xylan, starch, casein, tributyrin, and lignin) was also tested by agar diffusion method [19]. Among cellulase-positive isolates, an isolate with the highest cellulase activity (one with the largest halo-zone around the colony on flooding with both reagents) was selected for further processing.

### 2.4. Identification of the Isolate

Both phenotypic and molecular techniques were used for identification of the isolate. Phenotypic (morphological, cultural, and biochemical) tests were performed using standard techniques [20]. For the molecular identification, DNA was extracted through the lysis method [21]. The 16s rDNA was amplified using (fD1) 5′ AGAGTTTGATCCTGGCTCAG 3′ forward primer and (rP2) 5′ ACGGCTACCTTGTTACGACTT 3′ reverse primer, respectively [22].

The PCR product from 16s rDNA-based PCR was cleaned using a QIA quick PCR purification kit (Qiagen Inc., San Diego, CA, USA) and sequenced in an ABI 3500 XL automatic DNA sequencer following amplification in one direction with 16S primers using the BigDye Terminator Cycle Sequencing kit (Applied Biosystems, Inc., Palo Alto, CA, USA). The sequence similarity search was carried out using the BLAST program of the National Center of Biotechnology Information (NCBI). Closely related sequences were aligned in Mega X, and phylogenetic tree was constructed by a neighbor joining method with 100 bootstrap replications [23]. The 16s rDNA sequence can be retrieved from NCBI with GenBank accession number KY744361.1.

### 2.5. Production of Crude Enzyme

Production of cellulase was carried out in a basal medium containing CMC as a sole carbon source. The composition of medium was 10 g/L CMC, 2 g/L tryptone, 4 g/L KH_2_PO_4_, 4 g/L Na_2_HPO_4_, 0.2 g/L MgSO_4_.7H_2_O, 0.001 g/L CaCl_2_·2H_2_O, 0.004 g/L FeSO_4_·7H_2_O, and pH 7.0 [24]. Inoculated production medium was cultured at 60°C and 100 rpm for 24 hours, the culture broth was subsequently centrifuged at 5000 rpm at 4°C for 10 min, and the supernatant obtained was used as crude enzyme.

### 2.6. Cellulase Assay

Cellulase activity was determined based on concentration of reducing sugar produced during enzymatic reaction using 3′5 ′dinitro-salicylic acid (DNS) method [25]. Crude enzyme extract, 500 *μ*L, was mixed with 500 *μ*L substrate (1% CMC prepared in 50 mM sodium acetate buffer pH 5.0) [26] and incubated in a water bath at 60°C for 30 min followed by addition of 1 mL DNS reagent, boiled for 5 min and cooled. The absorbance was taken at 540 nm in UV spectrophotometer (6715 UV/Vis Spectrophotometer JENWAY). The supernatant from uninoculated media was used as the control. A standard curve was simultaneously drawn for estimating reducing sugars with glucose standards. The enzyme activity was expressed as enzyme units per mL (U/mL). One enzyme unit (U) was defined as the amount of enzyme that produced 1 *μ*mol of reducing sugar measured as glucose per mL per minute under assay conditions and the specific enzyme activity was measured as follows: specific enzyme activity = enzyme (U/mL)/protein concentration (mg/mL) [27]. The protein content of the enzyme samples was determined using Bradford assay following micro assay protocol using bovine serum albumin (BSA) as standard protein [28].

### 2.7. Optimization of Cellulase Production

Effect of various parameters like temperature, pH, media components, and other growth conditions was assessed for the optimum production of cellulase. During each optimization step, the previous optimum parameter obtained was used on the subsequent optimization of next parameter and optical density (OD) of the culture was measured at 600 nm to assess the growth of the organism. All the experiments were performed in triplicate.

#### 2.7.1. Temperature and Incubation Time

Four sets of flasks, each set having four pairs of flasks containing 50 mL cellulase production medium (an inoculated test flask and a control in each pair), were prepared, and each set was incubated at a temperature interval of 5°C from 50 to 65°C in shaking incubators at a speed of 100 rpm. From each set, a pair of flasks (one inoculated and one control) was taken out for measuring enzyme activity by DNS assay at 16, 20, 24, and 40 hours of incubation [29].

#### 2.7.2. pH

For the optimization of pH, different sets of media each containing test flasks and a control flask having a range of pH from 5.5 to 8.0 with 0.5 pH unit interval were prepared. The pH of each media was maintained with drop-wise addition of 1 N HCl and 1 N NaOH as required. Inoculum (0.1%) was added to each set of test flasks under sterile condition, and the flasks along with controls were incubated in a shaking incubator (Major Science, Taiwan) at 100 rpm for the optimum incubation time. DNS assay was performed to determine the optimum pH for maximum cellulase production [29, 30].

#### 2.7.3. N-Source and C-Source

Various organic nitrogen sources: yeast extract (YE), malt extract (ME), peptone, tryptone, and urea at the concentration of 0.2%, were used in the enzyme production media with previous parameters optimized. Further, the effect of various concentration of YE (0.02%-0.5%) on optimum production of enzyme was also determined [29]. Similarly, three different carbon sources: CMC, avicel, and cellobiose, in 1% concentration were incorporated in production media to determine the optimum production of enzyme. Again, to determine the optimum CMC concentration for maximum enzyme production, a range of CMC concentrations (0.5% to 2% with 0.5% interval) was used, and enzyme activity was measured using DNS assay [30].

### 2.8. Partial Purification of Crude Enzyme

All optimized parameters were applied in enzyme fermentation culture, and the crude enzyme was harvested from the culture broth as mentioned above. Crude enzyme thus obtained was subjected to salt precipitation (80% saturation of ammonium sulphate) and centrifuged at 16,000 g for 12 min. Resulting precipitate was dissolved in minimum amount of 50 mM Tris pH 7.0. The enzyme was then dialyzed (6-8 kDa size exclusion, SpectraPor, India) against the same buffer for 30 hours with 5 buffer changes during that interval [31]. Next, dialyzed enzyme was further purified on Sephadex G-75 column using 50 mM NaCl as the solvent front [32]. Thirty fractions of 1 mL were collected at a flow rate of 0.4 mL/min. Eluted fractions were monitored for protein concentration at 280nm and were assayed for enzyme activity. Fractions with high protein concentration and enzyme activity were pooled together and salt precipitated at 80% saturation. The precipitate was collected by centrifugation at 10,000 g and 4°C for 12 min, and it was redissolved in minimum amount of 50 mM Tris pH 7.0 and dialyzed against the same buffer as earlier. The concentrated enzyme thus obtained was stored at -20°C for further analysis. The specific activity of enzyme at each purification step was calculated using DNS and Bradford assays.

### 2.9. SDS-PAGE and Molecular Weight Determination

The molecular weight (MW) of the cellulase and the degree of purification were determined using Sodium dodecyl sulphate-polyacrylamide gel electrophoresis (SDS-PAGE). Enzyme samples (20 *μ*L each) were denatured by heating with loading dye (1 × final concentration) for 5 min at 95°C. The samples were cooled, loaded into 12% SDS PAGE gel along with broad range (6.5-116 kDa) protein marker (BIONEER, USA), and subsequently stained with Coomassie blue for visualization [33].

### 2.10. Characterization of Cellulase

The partially purified enzyme was used for biochemical characterization. Effect of different physicochemical parameters on enzyme activity was determined. To determine the effect of temperature/thermostability of the enzyme, 500 *μ*L aliquots of enzyme were incubated for an hour at 50, 60, 70, and 80°C. After incubation, 500 *μ*L substrate (1% CMC prepared in sodium acetate buffer of pH 5.0) was added to each tube, and the residual enzyme activity was measured using DNS assay. A reaction mixture without enzyme was used as a control. The effect of incubation time was determined by incubating the enzyme substrate mixture for 30, 60, 90, and 120 min followed by DNS assay. Similarly, the effect of pH on enzyme activity was determined by mixing 500 *μ*L of the enzyme with 500 *μ*L substrate prepared on buffers of various pH (1% CMC prepared in 50 mM CH_3_COOH-CH_3_COONa (pH 4.0-5.0), 50 mM Na_2_HPO_4_-NaH_2_PO_4_ (pH 6.0–pH 8.0) and 50 mM Glycine-NaOH (pH 9.0-11.0)) [34] followed by DNS assay. Finally, the effect of substrate concentration on enzyme activity was determined by mixing 500 *μ*L of the enzyme with 500 *μ*L of the substrate (CMC) of various concentrations (0.3%, 0.5%, 0.8%, 1%, 1.3%, 1.6%, and 2%) prepared on 50 mM Na_2_HPO_4_-NaH_2_PO_4_ buffer pH 6.0 followed by DNS assay.

Determining the effect of various metal ions involved the addition of various salt solutions (100 mM) prepared in 50 mM sodium phosphate buffer pH 6.0 to a final concentration of 10 mM to the reaction mixture followed by measurement of the amount of glucose produced in each case. Reaction mixture without any additive served as control. Different salts (additives) used were NaCl, FeSO_4_, MgSO_4_, CaCl_2_, ZnSO_4_, CoCl_2_, EDTA, Pb_3_O_4_, and CuSO_4_ [31]. Finally, the activity of enzyme on various substrates was measured by DNS assay of mixtures of enzyme with various substrates (CMC, avicel, cellobiose, xylan, and starch) prepared in optimum concentration (0.8%) and pH 6 [31].

### 2.11. Statistical Analysis

Statistical analysis was performed in Excel for mac Version 16.50. Error bars represent the standard error of the mean (SEM) calculated using the mean of the triplicate measurements and their standard deviation (SD). *T*-statistic was calculated, where applicable, using a two tailed *t*-test for unpaired sample assuming equal variance, and *p* value is represented as nonsignificant or “ns” for *p* > 0.05 and by the number of asterisks for significant results at significance level of *p* < 0.05 as indicated in the figure legend.

## 3. Results

### 3.1. Screening of Isolates for Extracellular Enzyme Production

Hot springs are one of the major sources for thermostable enzyme producing microorganisms. In Nepal, there are many hot springs which have fairly been explored for their microbial diversity and extracellular enzymes produced by those microorganisms. In this study, forty-four bacterial clones isolated from Kharpani hot spring water were first screened for cellulase activity. Out of forty-four isolates, KP43 was found to be a potent cellulose degrader with highest zone of hydrolysis by cell free culture filtrate. Thus, the isolate was selected for subsequent screening of other extracellular enzyme activities. Apart from cellulase, the isolate KP43 also showed xylanase, pectinase, caseinase, amylase, and lipase activities on agar plates incorporated with respective substrates, i.e., xylan, pectin, casein, starch, and tributyrin.

### 3.2. Identification of the Isolate KP43

The isolate was characterized by morphological observation, biochemical tests, and genetic analysis. The colony morphology characteristics were examined on 48 h culture on nutrient agar. The isolate was Gram positive (Figure 1(a)), motile, catalase, and oxidase-positive and endospore-producing bacillus. It was able to grow well within temperature range of 35-75°C with optimum growth observed at 60°C (Figure 1(b)). No growth was observed below 35°C and above 75°C. The phenotypic properties of the isolate KP43 are shown in Table 1.

Approximately 1.5 kb 16s rDNA was amplified from genomic DNA of isolate KP43 (Figure 1(c)) and sequenced. Similarity search of partial 16s rDNA gene sequence by BLAST showed maximum identity (99.93%) with strains of *Geobacillus kaustophilus* and *Geobacillus thermoleovorans* followed by those of *Geobacillus thermoparaffinivorans* and the genus *Bacillus*. A phylogenetic analysis was conducted in MEGA X. A phylogenetic tree constructed using 16s rDNA sequence demonstrated that the strain KP43 formed a cluster with *Geobacillus kaustophilus* NBRC 10224 (Figure 1(d)). The analysis involved six 16s rDNA nucleotide sequences of the different *Bacillus* species, obtained from NCBI GenBank (accession numbers shown in parenthesis). There were a total of 1305 positions in the final dataset. Based on these results and its phenotypic characteristics, the isolate was designated as *Geobacillus* sp. KP43. The partial 16s rDNA sequence of the isolate has been deposited in GenBank with accession number KY744361.1.

### 3.3. Enzyme Assays

#### 3.3.1. Optimization of Fermentation Condition for Cellulase Production

Different parameters affect the production of cellulase enzyme by microorganisms. The optimal fermentation condition for cellulase production was estimated by growing the bacterial isolate in the culture medium by varying the different parameters. The cellulase production was highly enhanced when CMC and yeast extract were used as carbon (Figure 2(a)) and nitrogen (Figure 2(b)) source, respectively.

The optimum cellulase activity was observed when the isolate was cultured in the medium having pH 6.5 (Figure 2(c)) supplemented with 0.04% yeast extract as N-source (Figure 2(d)) and 1% CMC as C-source (Figure 2(e)) at 55°C for 18 hours (Figure 2(f)). The enzyme production was slightly increased with the increase of CMC concentration from 0.5% to 1% and declined sharply thereafter (Figure 2(e)). Similar trend was observed for optimization of yeast extract concentration although the decrease in activity was not as sharp after 0.04% of YE as observed for CMC (Figure 2(d)).

#### 3.3.2. Partial Purification of Crude Enzyme

For the purification of cell free supernatant of *Geobacillus* sp. KP43 isolate, the crude enzyme was precipitated at 80% ammonium sulphate saturation which was then dialyzed with 50 mM phosphate buffer followed by Sephadex column chromatography. The protein concentration of crude enzyme, dialyzed product, and column purified enzyme was determined using Bradford assay.

Specific activity of enzyme was determined to be 0.186 U/mg, 0.19 U/mg, and 0.467 U/mg, respectively (Table 2). The molecular weight of the enzyme was found to be approximately 66 kDa as observed on 12% SDS-PAGE (Figure 3).

#### 3.3.3. Biochemical Characterization of Enzyme

Partially purified enzyme was used for its biochemical characterization, in which the optimum conditions of temperature, pH, duration of incubation with substrate, type and concentration of substrate, and the effect of various metal ions on enzyme activity were determined. The results obtained are presented in Figure 4.

The optimum incubation time for enzyme-substrate mix at 60°C was found to be 1 hour (Figure 4(a)), and the pH for the utmost activity of the partially purified enzyme was found to be 7 (Figure 4(c)). Cellulase from *Geobacillus* sp. KP43 exhibited its stability more than 50% within the pH range of 5 to 11 (Figure 4(c)), and maximal residual activity was observed at 70°C (Figure 4(b)) demonstrating its broad pH tolerance and excellent thermostability. The maximum residual activity at 70°C also indicates that the partially purified enzyme has optimum activity at this temperature. Beyond this temperature range, the activity/stability of the enzyme decreased sharply dipping close to 20% of maximal activity at 80°C. Regarding the substrate specificity, CMC was found to be the best substrate among other substrates like avicel, cellobiose, starch, and xylan for the partially purified enzyme, which showed its utmost activity at 0.8% CMC concentration (Figures 4(d) and 4(e)). Similarly, 10 mM concentration of different salts showed varied effects on partially purified cellulase activity (Figure 4(f)). The metal ion Fe^2+^ highly stimulated the cellulase activity by nearly fourfold while Na^+^ and Co^2+^ had no effect on the enzyme activity. Among the different salts tested, cellulase activity was almost completely inhibited by EDTA and Cu^2+^ ions and moderately, yet significantly (*t*-test), by rest of the ions such as Zn^2+^, Ca^2+^, Mg^2+^, and Pb^3+^ (Figure 4(f)).

## 4. Discussion

The cellulolytic microorganisms such as *Trichoderma*, *Aspergillus*, *Pellicularia*, *Penicillium*, *Acremonium*, and *Humicola* obtained from diverse environment were heat-sensitive [35]. Therefore, the hot spring water sample was chosen with the hope of isolating thermophiles that produce the thermostable cellulase. Among the cellulase positive isolates, one with the highest cellulase activity (ratio of zone diameter to colony diameter of 4.2) was selected for further processing. An isolate with colony or crude enzyme halo produced on a substrate that exceeds the colony diameter or well diameter by a factor of two or more are regarded as a polysaccharide-degrading enzyme producer [36].

Phenotypic tests give the preliminary idea of bacterial identity, but the information from 16s rDNA genotyping enables almost complete identification. The 16s rDNA has hypervariable regions where the sequences are diverged over evolutionary time [37]. However, conserved intervening regions enable primer binding and amplification of those hypervariable regions. The NCBI BLAST of partial 16s rDNA sequence produced the highest number of hits matching to *Geobacillus kaustophilus*, *Geobacillus thermoleovorans*, and other *Geobacillus* species. However, Ng et al. reported that the annotations of complete genome sequence of *Geobacillus kaustophilus* did not predict any *cellulase* homologous suggesting the isolate is more likely to be *Geobacillus thermoleovorans* [38]. Cellulolytic activity of *Geobacillus thermoleovorans* (strain T4) was reported earlier [39]. Furthermore, this species of *Geobacillus* was reported to be a sporing bacterium with terminal or subterminal endospores, catalase, and oxidase positive and having optimum growth temperature of 60°C and pH 6.0 to 7.0 [39, 40], in complete agreement with the results of this study. However, the taxonomy of *Geobacillus* is complicated [41], and further identification to confirm the species of the strain KP43 requires other elucidations such as fatty acid compositions, DNA-DNA hybridization kinetics, and morphology and physiology evaluations [38]. Hence, the isolate was simply designated as *Geobacillus* sp. KP43.

Additionally, other extracellular enzyme activities of the isolate agree with previous studies, which reported amylase, caseinase, and lipase activity on *Geobacillus thermoleovorans* [42, 43]. Although some studies have reported the absence of complete cellulase system in bacteria of *Bacillus* genus with their activity primarily focused on CMC and none on avicel [27, 44], isolate in this study seems to have moderate activities against CMC, avicel, and cellobiose. Nonetheless, exoglucanase activity (on avicel) in certain bacilli has been reported earlier [45]. Since the bacterium grows well in thermophilic range, the extracellular enzymes produced by it are thermotolerant with potentials to be used in harsh industrial settings. This suggests the isolate to be a good source of variety of enzymes of industrial importance.

Optimization of cellulase production indicated that a medium containing 1% CMC, 0.04% yeast extract and pH 6.5 was optimal for cellulase production at 55°C for 18 hours. Although optimizing a parameter at once, as used in this study, has long been used in the field, modern statistical/mathematical techniques that allow the simultaneous determination of the effect of multiple independent parameters on enzymatic saccharification are being increasingly used for optimization of bioprocesses recently. In this regard, response surface methodology (RSM) has widely been used for optimization of fermentation medium for maximum saccharification using microbes derived from various sources [46–51]. However, artificial neural network (ANN) using Box-Behnken design was reported to be somewhat superior to RSM for optimization of wheat straw saccharification by *Trichoderma viride* [52].

Following enzyme production, its purification steps such as salt precipitation, dialysis, and Sephadex G-75 column chromatography were carried out to make the characterization of enzyme more reliable. The specific activity of the enzyme increased in each purification step as expected, which might be reflecting the loss of an unwanted fraction of crude enzyme at each step. Indeed, the purification process ensured the higher purity of the enzyme in subsequent steps as indicated by its improved specific activity. This trend is in agreement with similar studies on *Bacillus subtilis* [31] and *Bacillus licheniformis* [27]. The 12% SDS-PAGE analysis revealed a prominent band of size approximately 66 kDa, which falls within a range of molecular mass of cellulase 31 to 94 kDa reported previously [53]. However, the size of endoglucanase “CelA” in *Geobacillus* sp. 70PC53 was reported as 43 kDa [38], and that of *Cellulomonas* sp. and *Bacillus megaterium* was reported to be approximately 53.55 kDa [54, 55].

While determining the activity and stability of enzyme at different temperature, the residual activity of enzyme after incubation for an hour at different temperatures was found highest at 70°C, which is in complete agreement with the previously reported optimal temperatures for cellulase from *Geobacillus* strain [56] and *Geobacillus thermoleovorans* T4 [39]. Moreover, cellulase from *Geobacillus thermoleovorans* T4 was stable for an hour at 70°C with more than 90% of activity retained [39] and endoglucanse from *Geobacillus* sp. 70PC53 was stable for 6 hours at 65°C [38]. Similarly, the optimum incubation time with substrate was found to be 1 hour, which indicates that an hour is the optimum time for formation of maximum enzyme-substrate complexes under the reaction conditions, which might vary under different settings.

The optimum pH for the enzyme activity was found to be 7.0, though the enzyme activity was comparable in pH range of 5.0 to 9.0. This was also reflected in the plate assay using Dingle's cup technique [57] with largest halozone at pH 6.5 in comparison to the halozone at pH 6.0 or 7.0 (data not shown). However, the optimum pH for endoglucanse [38] and cellulase [56] from *Geobacillus* sp. was reported to be 5.0. Indeed, the enzyme seems to be affected less by pH as it remained active over a pH range of 5.0 to 11.0 and maintained the similar level of activity between pH 5.0 to 9.0. Ng and colleagues also reported that endoglucanse from *Geobacillus* sp. 70PC53 was stable for up to 16 hours at pH range of 5.0 to 9.0, with loss of only 20% enzyme activity [38].

Metal ion Fe^2+^ seems to stimulate the enzyme activity remarkably at 10 mM final concentration with 345% increase over the control. Different metal ions added with purified enzyme may act as cofactors or as inhibitors. This seems to be dependent on the concentration of metal ions used as suggested by reports [38, 58]. The inhibitory effect of Cu^2+^ and Zn^2+^ at this concentration was also reported elsewhere [38]. Similarly, activity of cellulase from *Geobacillus* sp. PW11 and PW13 was reported to be increased by 2.5 and 2.4 folds, respectively, in the presence of 10 mM Fe^2+^ as reported here. However, other divalent cations—Ca^2+,^ Mg^2+,^ Zn^2+,^ and Hg^2+^—were reported to have no effect unlike in this study [59].

The activity of enzyme tested with different substrates showed the highest activity against CMC, followed by starch, xylan, and cellobiose with the least activity against avicel. This tells us that the organism is potent in terms of enzyme production and agrees with preliminary extracellular enzyme screening results. The presence of all three enzyme specificities, i.e., endoglucanse, exoglucanase, and cellobiase, suggests the presence of complete cellulase enzyme system in *Geobacillus* sp. KP43 unlike in other members of genus *Bacillus* as reported earlier [27, 44]. Regarding substrates, many studies frequently use raw (ligno-)cellulosic substrates as C-source instead of synthetic substrates, which can be preferable in the sense that these raw substrates are more representative of the inherent complexity of natural lignocellulosic materials. For instance, five species of *Bacillus* and *Pseudomonas stutzeri* showed maximum cellulase production using eucalyptus leaves as C-source among others such as corncob, sugarcane bagasse, rice husk, wheat straw, and seed pod of *Bombax ceiba* [60]. Similarly, the order of enzyme production using *Bacillus subtilis* strain with various substrates was sugarcane bagasse>wheat straw>rice husk, wheat bran>soybean meal>corncobs [61].

The enzymatic capabilities of *Geobacillus* sp. KP43 reported in this study are in agreement with the previous studies reporting high biotechnological potential of the *Geobacillus* sp. producing thermostable enzymes such as cellulases [39], xylanases [62, 63], proteases [64], and amylases and lipases [65, 66]. Follow-up studies can be focused on improving the cellulolytic potential and scaling up the production of the cellulase by genetic and/or metabolic engineering strategies. For instance, a recombinant glycoside hydrolase enzyme expressed in *Escherichia coli* BL21, derived originally from hyperthermophile *Thermotoga maritima* MSB8, retained its thermostability at 80°C for 72 hours [67]. Furthermore, metabolic engineering of cellulolytic microbes to enhance the bioethanol production can be another strategy to improve the utility of potent microbial strains with industrial applications [68–70]. This approach was also adopted more recently in *Corynebacterium glutamicum* for hydrocarbon biofuel production from lignocellulosic biomass [71].

## 5. Conclusion

A thermophilic bacterium *Geobacillus* sp. KP43 was isolated, and cellulase enzyme it produced was partially purified and characterized. This is the first report on characterization of thermostable cellulase from *Geobacillus* sp. isolated from Kharpani hot spring, Nepal. The thermophilic bacterium, also producing extracellular enzymes like xylanase, amylase, lipase, and protease besides thermoalkaliphilic cellulases, is suitable for diverse applications from waste management to biofuel production. Future studies can be focused on scaling up of enzyme production by heterologous expression of cellulase gene in *Escherichia coli*, further purification of the enzyme, and the pilot scale bioethanol production.

## Figures and Tables

**Figure 1:** Characterization of the isolate *Geobacillus* sp. KP43. (a) Gram staining of the organism (Gram-positive long rods). (b) Growth curve of the organism over a temperature range of 35 to 80°C shows optimum growth at 60°C. (c) 16s rDNA amplification showing an amplicon of ~1.5 kb (lane 1; L: DNA ladder). (d) Phylogenetic relation of *Geobacillus* sp. KP43 with different bacilli from the NCBI Genebank database based on 16s rDNA gene sequence. The gene bank accession numbers of respective strains are given in parentheses. The tree diagram was generated by the neighbor joining method using Mega X.

**Figure 2:** Effect of various parameters on growth and cellulase enzyme production by isolate *Geobacillus* sp. KP43. Effects of Carbon source (a), nitrogen source (b), pH (c), yeast extract (YE) concentration (d), CMC concentration (e), and incubation time and temperature (f) are shown. Error bars represent the mean ± SEM of respective triplicate measurements [SEM: standard error of the mean].

**Figure 3:** SDS-PAGE of cellulase enzyme extracted from *Geobacillus* sp. strain KP43 (1 = cell pellet, 2 = crude enzyme, 3 = precipitated enzyme, 4 = dialyzed product, 5 = column purified enzyme, and M = protein marker).

**Figure 4:** Effect of incubation time (a), temperature (b), pH (c), substrates (d), CMC concentration (e), and different salts at 10 nM (f) on cellulase activity. Error bars represent mean ± SEM from respective triplicate measurements. Effect of different salts (f) is tested against control (no salt condition) using a two-tailed *t*-test, and the *p* value is represented as “asterisk(s)” or “ns” above the respective bars [^ns^*p* > 0.05 (nonsignificant), ^∗^*p* < 0.05,  ^∗∗^*p* < 0.01,  ^∗∗∗^*p* < 0.001, and^∗∗∗∗^*p* < 0.0001; SEM: standard error of the mean].

**Table 1:** Morphological and physiological properties of isolate KP43.

Tests	Results
Gram staining	Gram-positive thin rods
Shape	Thin rod
Catalase test	Catalase positive
Oxidase test	Oxidase positive
Motility test	Motile
Growth range (temperature)	Growth seen between 35 and 75°C
Optimum temperature	60°C
Capsule staining	Noncapsulated
Spore staining	Spore bearer with terminal endospore in nonswollen sporangia

**Table 2:** Activity of cellulase enzyme at different purification steps.

Enzyme	Activity (U/mL)	Protein content (mg/mL)	Specific activity (U/mg)	Purification fold
Crude	0.010	0.051	0.186	1
Salt precipitated and dialyzed	0.024	0.128	0.190	1.021
Column purified	0.026	0.055	0.467	2.488

## Data Availability

The data used to support the findings of this study are included within the article.

## References

[1] Rampelotto P. H. (2013). Extremophiles and extreme environments. *Life*.

[2] van den Burg B. (2003). Extremophiles as a source for novel enzymes. *Current Opinion in Microbiology*.

[3] Amjad K. (2011). Isolation and characterization of three thermophilic bacterial strains (lipase, cellulose and amylase producers) from hot springs in Saudi Arabia. *African Journal of Biotechnology*.

[4] Kristjansson J. K. (1991). *Thermophilic bacteria*.

[5] Adams M. W., Kelly R. M. (1998). Finding and using hyperthermophilic enzymes. *Trends in Biotechnology*.

[6] Liszka M. J., Clark M. E., Schneider E., Clark D. S. (2012). Nature versus nurture: developing enzymes that function under extreme conditions. *Annual Review of Chemistry, Biomolecular Engineering*.

[7] Kuhad R. C., Gupta R., Singh A. (2011). Microbial cellulases and their industrial applications. *Enzyme Research*.

[8] Wyman C. E. (2007). What is (and is not) vital to advancing cellulosic ethanol. *Trends in Biotechnology*.

[9] Turner B. T., Plevin R. J., O'Hare M., Farrell A. E. (2007). *Creating markets for green biofuels: measuring and improving environmental performance*.

[10] Balat M., Balat H. (2009). Recent trends in global production and utilization of bio-ethanol fuel. *Applied Energy*.

[11] Patel A. K., Singhania R. R., Sim S. J., Pandey A. (2019). Thermostable cellulases: current status and perspectives. *Bioresource Technology*.

[12] Vaishnav N., Singh A., Adsul M. (2018). _Penicillium_ : the next emerging champion for cellulase production. *Bioresource Technology Reports*.

[13] Meyer-Dombard D. R., Shock E. L., Amend J. P. (2005). Archaeal and bacterial communities in geochemically diverse hot springs of Yellowstone National Park, USA. *Geobiology*.

[14] Ranjit M. Geothermal Energy Update of Nepal.

[15] Yadav P., Korpole S., Prasad G. S. (2018). Morphological, enzymatic screening, and phylogenetic analysis of thermophilic bacilli isolated from five hot springs of Myagdi Nepal. *Journal of Applied Biology & Biotechnology*.

[16] Mg Z. L. M., Than W. M., Myint M. (2015). Study on the cellulase enzyme producing activity of bacteria isolated from manure waste and degrading soil. *International Journal of Technical Researcj amd Applications*.

[17] Kasana R. C., Salwan R., Dhar H., Dutt S., Gulati A. (2008). A rapid and easy method for the detection of microbial cellulases on agar plates using Gram’s iodine. *Current Microbiology*.

[18] Teather R. M., Wood P. J. (1982). Use of Congo red-polysaccharide interactions in enumeration and characterization of cellulolytic bacteria from the bovine rumen. *Applied and Environtal Microbiology.*.

[19] Samad M. Y. A., Razak C. N. A., Salleh A. B., Zin Wan Yunus W. M., Ampon K., Basri M. (1989). A plate assay for primary screening of lipase activity. *Journal of Microbiological Methods*.

[20] Benson H. J. (2002). *Microbiological applications: Laboratory Manual in General Microbiology. Eighth Edition ed*.

[21] Ceron J., Ortíz A., Quintero R., Güereca L., Bravo A. (1995). Specific PCR primers directed to identify cryI and cryIII genes within a Bacillus thuringiensis strain collection. *Applied and Environtal. Microbiology.*.

[22] Weisburg W. G., Barns S. M., Pelletier D. A., Lane D. J. (1991). 16S ribosomal DNA amplification for phylogenetic study. *Journal of Bacteriology*.

[23] Kumar S., Stecher G., Li M., Knyaz C., Tamura K. (2018). MEGA X: molecular evolutionary genetics analysis across computing platforms. *Molecular Biology and Evolution*.

[24] Ray A. K., Bairagi A., Ghosh K. S., Sen S. K. (2007). Optimization of fermentation conditions for cellulase production by Bacillus subtilis CY5 and Bacillus circulans TP3 isolated from fish gut. *Acta Ichthyologica et Piscatoria*.

[25] Miller G. L. (1959). Use of dinitrosalicylic acid reagent for determination of reducing sugar. *Analytical Chemistry*.

[26] Sadhu S., Saha P., Sen S. K., Mayilraj S., Maiti T. K. (2013). Production, purification and characterization of a novel thermotolerant endoglucanase (CMCase) from Bacillus strain isolated from cow dung. *Springer Plus*.

[27] Bischoff K. M., Rooney A. P., Li X. L., Liu S., Hughes S. R. (2006). Purification and characterization of a family 5 endoglucanase from a moderately thermophilic strain of Bacillus licheniformis. *Biotechnology Letters*.

[28] Kruger N. J. (2009). The Bradford method for protein quantitation. *The Protein Protocols Handbook*.

[29] Abol Fotouh D. M., Bayoumi R. A., Hassan M. A. (2016). Production of thermoalkaliphilic lipase from Geobacillus thermoleovorans DA2 and application in leather industry. *Enzyme Research*.

[30] Gautam S. P., Bundela P. S., Pandey A. K., Khan J., Awasthi M. K., Sarsaiya S. (2011). Optimization for the production of cellulase enzyme from municipal solid waste residue by two novel cellulolytic fungi. *Biotechnology Research International*.

[31] Yin L.-J., Lin H.-H., Xiao Z.-R. (2020). Purification and characterization of a cellulase from Bacillus subtilis YJ1. *Journal of Marine Science and Technology*.

[32] Singh V., Kumar A. (1998). Production and purification of an extracellular cellulase from Bacillus brevis vs-1. *IUBMB Life*.

[33] Laemmli U. K. (1970). Cleavage of structural proteins during the assembly of the head of bacteriophage T4. *Nature*.

[34] Lin L., Kan X., Yan H., Wang D. (2012). Characterization of extracellular cellulose-degrading enzymes from Bacillus thuringiensis strains. *Electronic Journal of Biotechnology*.

[35] Fujimoto N., Kosaka T., Nakao T., Yamada M. (2011). Bacillus licheniformis bearing a high cellulose-degrading activity, which was isolated as a heat-resistant and micro-aerophilic microorganism from bovine rumen. *The Open Biotechnology Journal*.

[36] Ten L. N., Im W. T., Kim M. K., Kang M. S., Lee S. T. (2004). Development of a plate technique for screening of polysaccharide-degrading microorganisms by using a mixture of insoluble chromogenic substrates. *Journal of Microbiological Methods*.

[37] Woese C. R. (1987). Bacterial evolution. *Microbiological Reviews*.

[38] Ng I.-S., Li C. W., Yeh Y. F. (2009). A novel endo-glucanase from the thermophilic bacterium Geobacillus sp. 70PC53 with high activity and stability over a broad range of temperatures. *Extremophiles*.

[39] Tai S.-K., Lin H.-P. P., Kuo J., Liu J.-K. (2004). Isolation and characterization of a cellulolytic Geobacillus thermoleovorans T4 strain from sugar refinery wastewater. *Extremophiles*.

[40] Dinsdale A. E., Halket G., Coorevits A. (2011). Emended descriptions of Geobacillus thermoleovorans and Geobacillus thermocatenulatus. *International Journal of Systematic and Evolutionary Microbiology*.

[41] Nazina T. N., Sokolova D. S., Grigoryan A. A. (2005). _Geobacillus jurassicus_ sp. nov., a new thermophilic bacterium isolated from a high-temperature petroleum reservoir, and the validation of the _Geobacillus_ species. *Systematic and Applied Microbiology*.

[42] Romano I., Poli A., Lama L., Gambacorta A., Nicolaus B. (2005). Geobacillus thermoleovorans subsp. stromboliensis subsp. nov., isolated from the geothermal volcanic environment. *Applied Microbiology*.

[43] Mahdhi A., Hmila Z., Behi A., Bakhrouf A. (2011). Preliminary characterization of the probiotic properties of Candida famata and Geobacillus thermoleovorans. *Iranian Journal of Microbiology*.

[44] Robson L. M., Chambliss G. H. (1984). Characterization of the cellulolytic activity of a Bacillus isolate. *Applied and Environtal Microbiology.*.

[45] Mawadza C., Hatti-Kaul R., Zvauya R., Mattiasson B. (2000). Purification and characterization of cellulases produced by two _Bacillus_ strains. *Journal of Biotechnology*.

[46] Tabssum F., Irfan M., Shakir H. A., Qazi J. I. (2018). RSM based optimization of nutritional conditions for cellulase mediated Saccharification by Bacillus cereus. *Journal of Biological Engineering*.

[47] Irfan M., Bakhtawar J., Shakir H. A., Khan M., Ali S. (2019). Utilization of peanut shells as substrate for cellulase production in submerged fermentation through Box-Behnken design. *International Journal of Biology and Chemistry*.

[48] Ghazanfar M., Irfan M., Tabssum F., Shakir H. A., Qazi J. I. (2018). Effect of different pretreatment conditions on Saccharum spontaneum for cellulase production by B. subtilis K-18 Through Box–Bhenken design. *Iranian Journal of Science and Technology, Transactions A: Science*.

[49] Irfan M., Mushtaq Q., Tabssum F., Shakir H. A., Qazi J. I. (2017). Carboxymethyl cellulase production optimization from newly isolated thermophilic Bacillus subtilis K-18 for saccharification using response surface methodology. *AMB Express*.

[50] Khalid S., Irfan M., Shakir H. A., Qazi J. I. (2017). Endoglucanase producing potential of bacillus species isolated from the gut of Labeo rohita. *Journal of Marine Science and Technology*.

[51] Majeed H. S., Irfan M., Shakir H. A., Qazi J. I. (2016). Filter paper activity producing potential of Aeromonas species isolated from the gut of Labeo rohita. *Pakistan Journal of Zoology*.

[52] Nelofer R. (2021). Conversion of wheat straw into fermentable sugars using carboxymethyl cellulase from trichoderma viride through Box-Behnken design and artificial neural network. *Journal of Microbiology, Biotechnology and Food Sciences*.

[53] Endo K., Hakamada Y., Takizawa S. (2001). A novel alkaline endoglucanase from an alkaliphilic Bacillus isolate: enzymatic properties, and nucleotide and deduced amino acid sequences. *Applied Microbiology and Biotechnology*.

[54] Bai H., Irfan M., Wang Y., Wang H., Han X. (2017). Purification and characterization of cellulose degrading enzyme from newly isolated cellulomonas sp. *Cellulose Chemistry and Technology*.

[55] Shahid Z., Irfan M., Nadeem M., Syed Q., Qazi J. I. (2016). Production, purification, and characterization of carboxymethyl cellulase from novel strain Bacillus megaterium. *Environmental Progress & Sustainable Energy*.

[56] Rastogi G., Bhalla A., Adhikari A. (2010). Characterization of thermostable cellulases produced by _Bacillus_ and _Geobacillus_ strains. *Bioresource Technology*.

[57] Dingle J., Reid W. W., Solomons G. L. (1953). The enzymic degradation of pectin and other polysaccharides. II—application of the ‘Cup-plate’ assay to the estimation of enzymes. *Journal of the Science of Food and Agriculture*.

[58] Phan M. T. T., Nguyen V. Q., le H. G., Nguyen T. K., Tran M. D. (2012). Molecular cloning gene and nucleotide sequence of the gene encoding an endo-1, 4-beta-glucanase from bacillus sp VLSH08 strain applying to biomass hydrolysis. *Journal of Vietnamese Environment*.

[59] Sharma P., Gupta S., Sourirajan A., Dev K. (2015). Characterization of extracellular thermophillic cellulase from thermophilic Geobacillus sp. isolated from Tattapani Hot spring of Himachal Pradesh, India. *International Journal of Advanced Biotechnology and Research*.

[60] Ghazanfar M., Irfan M., Nadeem M. (2021). Isolation of cellulolytic bacteria from soil and valorization of different lignocellulosic wastes for cellulase production by submerged fermentation. *Cellulose Chemistry and Technology*.

[61] Mohsin Arshad M. I., Asad-Ur-Rehman M. N., Zile Huma H. A. S. (2017). Optimization of medium and substrate for CMCase production by Bacillus subtilis-BS06 in submerged fermentation and its applications in saccharification. *Punjab University Journal of Zoology*.

[62] Liu J.-R., Duan C. H., Zhao X., Tzen J. T. C., Cheng K. J., Pai C. K. (2008). Cloning of a rumen fungal xylanase gene and purification of the recombinant enzyme via artificial oil bodies. *Applied Microbiology and Biotechnology*.

[63] Sharma A., Adhikari S., Satyanarayana T. (2007). Alkali-thermostable and cellulase-free xylanase production by an extreme thermophile Geobacillus thermoleovorans. *World Journal of Microbiology and Biotechnology*.

[64] Chen X.-G., Stabnikova O., Tay J. H., Wang J. Y., Tay S. T. L. (2004). Thermoactive extracellular proteases of Geobacillus caldoproteolyticus, sp. nov., from sewage sludge. *Extremophiles*.

[65] Abdel-Fattah Y. R., Gaballa A. A. (2008). Identification and over-expression of a thermostable lipase from _Geobacillus thermoleovorans_ Toshki in _Escherichia coli_. *Microbiological Research*.

[66] Leow T. C., Rahman R. N. Z. R. A., Basri M., Salleh A. B. (2007). A thermoalkaliphilic lipase of Geobacillus sp. T1. *Extremophiles*.

[67] Mustafa M., Ali L., Islam W. (2022). Heterologous expression and characterization of glycoside hydrolase with its potential applications in hyperthermic environment. *Saudi Journal of Biological Sciences*.

[68] Su H., Lin J., Wang G. (2016). Metabolic engineering of _Corynebacterium crenatium_ for enhancing production of higher alcohols. *Scientific Reports*.

[69] Song X., Li Y., Wu Y. (2018). Metabolic engineering strategies for improvement of ethanol production in cellulolytic Saccharomyces cerevisiae. *FEMS Yeast Research*.

[70] Li J., Zhang Y., Li J., Sun T., Tian C. (2020). Metabolic engineering of the cellulolytic thermophilic fungus Myceliophthora thermophila to produce ethanol from cellobiose. *Biotechnology for Biofuels and Bioproducts*.

[71] Xu Y. Y., Hua K. J., Huang Z. (2022). Cellulosic hydrocarbons production by engineering dual synthesis pathways in Corynebacterium glutamicum. *Biotechnology for Biofuels and Bioproduct*.

